The article "A Method of CT Image Denoising Based on Residual Encoder-Decoder Network" was published in 2021. Journal: J Healthc Eng.

# A Method of CT Image Denoising Based on Residual Encoder-Decoder Network

**DOI:** 10.1155/2021/2384493

**Published:** 2021-09-23

**Authors:** Yali Liu

**Affiliations:** Faculty of Economics and Management, Shangluo University, Shaanxi, Shangluo 726000, China

## Abstract

Low-dose computed tomography (CT) has proved effective in lowering radiation risk for the patients, but the resultant noise and bar artifacts in CT images can be a disturbance for medical diagnosis. The difficulty of modeling statistical features in the image domain makes it impossible for the existing methods that directly process reconstructed images to maintain the detailed texture structure of images while reducing noise, which accounts for the failure in CT diagnostic images in practical application. To overcome this defect, this paper proposes a CT image-denoising method based on an improved residual encoder-decoder network. Firstly, in our approach, the notion of recursion is integrated into the original residual encoder-decoder network to lower the algorithm complexity and boost efficiency in image denoising. The original CT images and the postrecursion result graph output after recursion are used as the input for the next recursion simultaneously, and the shallow encoder-decoder network is recycled. Secondly, the root-mean-square error loss function and perceptual loss function are introduced to ensure the texture of denoised CT images. On this basis, the tissue processing technology based on clustering segmentation is optimized considering that the images after improved RED-CNN training will still have certain artifacts. Finally, the experimental results of the TCGA-COAD clinical data set show that under the same experimental conditions, our method outperforms WGAN in average postdenoising PSNR and SSIM of CT images. Moreover, with a lower algorithm complexity and shorter execution time, our method is a significant improvement on RED-CNN and is applicable for actual scenarios.

## 1. Introduction

The high radiation technology dose to the human body continues to develop in the computed tomography (CT) scanning process, and CT images have seen ever-wider application in medical diagnosis [1, 2]. By cutting X-ray tube current, low-dose scanning requires less radiation dose and therefore lowers the signal-to-noise ratio in projection data. Noise and artifacts are blended into CT images reconstructed by the filtered back projection (FBP) algorithm, which affects the accuracy of subsequent clinical diagnosis. Therefore, studying how to reconstruct the reconstructed CT image from original noisy projection data is of great significance and practical value [3].

At this stage, the methods of improving the quality of low-dose CT (LDCT) images can be divided into projection domain denoising algorithm [4], image reconstruction algorithm [5], and image domain denoising algorithm [6]. These image-denoising methods, however, prove ineffective in improving CT image quality. Furthermore, it is difficult to describe these methods with a precise model since they have a large number of iterations and take a long time, and the distribution of image noise after processing becomes complicated. And there may be artifacts in images. Thus, the traditional image-denoising methods can hardly attain the desired effects. Thus, it is difficult to achieve the desired effects with traditional image denoising methods. The traditional methods can suppress noise and artifacts, but they are prone to the loss of edge and detailed information. Therefore, the resultant denoised CT images cannot meet the actual clinical diagnosis application [7].

The rapid development of deep neural networks offers new insights into how to address the problem in LDCT image denoising [8, 9]. Because of the powerful feature learning and mapping capabilities of deep neural networks, deep neural networks show better reconstruction quality and faster speed than traditional methods. To date, the deep neural network has achieved good results in LDCT image denoising. However, since these networks use mean square error (MSE) as loss function, minimizing MSE usually incurs detail and loss and excessive edge smoothness. At the same time, the image texture that is important to the human eye perception is ignored [10].

We, therefore, propose RED-CNN, a CT image-denoising algorithm based on residual encoder-decoder (RED) convolutional neural network, namely, RED-CNN. Using sampling operations to learn end-to-end nonlinear mapping in a multiscale space, our method is able to reconstruct the denoised images directly. At the same time, convolution and deconvolution operations are used to better extract features and restore the details of CT images. The main innovations of the paper are as follows:

1. The proposed CT image-denoising method based on an improved RED network uses the same shallow RED network to recursively construct a new network, thereby reducing network complexity.
2. In order to improve the visual artifacts of CT images after denoising, a new joint loss is proposed by combining the advantages of MSE loss function and perceptual loss function, which can better reconstruct the details and texture of images.
3. Residual learning is combined with traditional optimization processing techniques. Introducing distance images into water images can help reduce data inconsistency and better improve the denoising effect of CT images.

## 2. Related Work

As a noninvasive imaging technique, computed tomography is widely used in industry, medicine, and many other fields. Of all the image reconstruction methods applied in X-ray CT imaging, FEP is the most widely used one. Generally, a good image can be reconstructed when the projection data is complete [11, 12].

The projection domain filtering algorithm filters the original data in the projection domain and then uses FBP to reconstruct CT images. Typical methods include bilateral filtering method [13], adaptive convolution filtering method [14], penalty weighted least square (PWLS) method [15], and so on.

Both the projection domain denoising algorithm and image reconstruction algorithm need to use projection data. In practical applications, however, projection data is usually used as an intermediate result of a CT scanner and is not accessible to ordinary users. As a method not reliant on projection data, the image domain denoising algorithm is able to denoise reconstructed CT images directly. It, therefore, has become a research hotspot in the field of LDCT image denoising [16–18]. In accordance with the theory that image data can be decomposed into information and time uncorrelated noise, reference [19] proposed a CT image-denoising method based on wavelet transformation. It could use the average and weighted wavelet coefficients of input images to reconstruct final denoising images. Reference [20] combined 3D filter with blind source separation (BSS) to extract noise statistics from noise components. A denoising method for CT images based on BSS for multiframe low-dose image sequences was proposed. Reference [21] proposed an improved SNCSR model and used the improved total variation (ITV) model to preprocess images. Aiming at the fringe artifacts in CT images, reference [22] proposed an image denoising algorithm based on discriminative weighted nuclear norm minimization (D-WNNM). The local entropy of images was used to distinguish fringe artifacts and organizational structure, and the weight coefficient of the weighted nuclear norm minimization (WNNM) denoising method was adaptively adjusted.

For its ability to extract features and map, deep learning is now widely used in image processing, and this method has greater advantages over traditional ones in removing complex noise from LDCT images. Reference [23] proposed a CT image denoising method based on generative adversarial network (GAN). By integrating visual perception into image denoising, this method reduces image noise while retaining relevant key information. Reference [24] incorporated structural similarity index into the GAN model and introduced a least square loss function penalty term to constrain CT images and further maintaining the texture detail and sharpness of CT images.

Although the projection domain denoising algorithm can make full use of statistical law for noise distribution in the projection domain, data inconsistencies may occur in the process of noise reduction in the projection domain. It is easy to introduce new noise or artifacts into reconstructed images, and the traditional single image denoising method cannot achieve desired effects [25]. Although the CT image denoising method based on deep learning can greatly remove the stripe artifacts and reduce the noise of CT images, the peak signal-to-noise ratio has been improved. However, the upsampling and downsampling links in network structure and methods based on MSE or weighted MSE are prone to cause loss of image details in the process of image denoising. In addition, the complex network structure model showed greater instability during the training process, and the network is difficult to converge [26, 27]. The RED-CNN is simple in structure, and continuously deepening the network structure can achieve effective denoising of CT images in complex and multinoise scenarios. For example, reference [28] proposed an image denoising method based on RED-CNN. The best denoising effect has been achieved in the objective evaluation index.

Based on easy expansion and strong adaptability of the RED-CNN deep neural network, this paper also proposes a new CT image denoising method combined with the recursive notion of network structure model. This method can better extract and recognize the feature information of images and use the same network structure to recursively construct a new network. By reducing the number of layers and convolution kernels in the RED network, the network complexity is lowered to achieve rapid denoising of CT images. On this basis, the principle of *k*-means clustering segmentation is integrated. CT images are optimized based on the threshold, which improves the details and texture of denoised images.

The remainder of this paper is arranged as follows.  Section 3 introduces CT image denoising model based on the improved RED network and its corresponding network structure model in detail.  Section 4 presents the experimental analysis of CT images in the TCGA-COAD clinical data set to verify the effectiveness of the proposed method. This paper is summarized in Section 5.

## 3. RED Network-Based CT Image Denoising

This section introduces the denoising model, network structure of RED-CNN, overall structure of recursive network, and the image optimization process after the RED-CNN model. Besides, root MSE and perceptual loss function are used as the loss functions of the overall network, which can partially address the problem of detail loss and preserve the image texture as well. Finally, the image optimization process after the RED-CNN model is introduced.

### 3.1. Noise Reduction Model

Assuming *x* ∈ R^*N×N*^ is normal-dose CT (NDCT) image, and *x* ∈ R^*N×N*^ is LDCT image. The purpose of CT image denoising is to map *z* to *x* by finding a suitable function *G*, which can be expressed as follows:

(1) $$\begin{array}{c} G:z⟶x, \end{array}$$

where *x* ∈ *R*^*N* × *N*^ is the sample of CT image distribution *P*_*r*_ under normal dose and *x* ∈ *R*^*N* × *N*^ is the sample of LDCT image distribution *P*_*L*_. The function *G* maps LDCT image distribution *P*_*L*_ to a specific image distribution *P*_*g*_ and make the generated distribution *P*_*g*_ as close as possible to the real sample distribution *P*_*r*_.

### 3.2. Network Structure

Figure 1 shows the overall structure of constructed image denoising network based on a shallow RED network. The RED network consists of 8 layers, with 4 of them being convolutional layers and the remainders deconvolutional layers arranged symmetrically. Each of the first 7 hidden layers has 64 convolution kernels, and the last layer is 1 convolution kernel.

In the overall network structure, the shallow encoder-decoder network in Figure 2 is recycled to generate the final denoising image. The specific notion is as follows: in each recursion, the original CT image and the result image output after the *s* recursion are simultaneously used as the input for the next recursion. It can avoid the loss of original image features in the recursive process, better extract the features of original input images, and retain the detailed information of images.

The recursive process of the network can be expressed as follows:

(2) $$\begin{array}{c} I_{1}=X,\\ O_{s}=F_{\text{RED}-\text{Net}}\left(I_{s}\right),\;1\leq s<S,\\ I_{s+1}=f_{\text{in}}\left(O_{s},X\right),\;1\leq s<S, \end{array}$$

where *S* represents the number of recursions, *X* represents the network input, RED-Net is the shallow RED network, *O*_*s*_ is the denoising CT image obtained from the *s* recursion, *f*_in_ represents the cascade operation between output *O*_*s*_ of the *s* recursion and original LDCT image, and *X*. *I*_*s* + 1_ is the input of the *s* + 1 recursion.

### 3.3. Loss Function

In conventional learning-based image reconstruction methods, root MSE is usually used as the objective function. The pixel-by-pixel comparison method can achieve a high signal-to-noise ratio, but the partial loss of detailed information tends to blur the image denoising results. Perceptual loss based on feature comparison is more in line with real visual perception and can help restore clearer images. However, pixel space, when covered evenly, can sometimes generate subtle visual artifacts.

A new joint loss is proposed so as to better reconstruct the details and image texture, a combination of both advantages.

(3) $$\begin{array}{c} L_{\text{Joint}}=L_{\text{MSE}}+L_{\text{Per}}, \end{array}$$

where *L*_MSE_ and *L*_Per_ represent the loss function of pixel-by-pixel comparison and semantic feature comparison, respectively.

(1) MSE loss function. The pixel-by-pixel loss function uses the traditional MSE method to calculate root MSE between denoised CT images and real images through pixel-by-pixel comparing and matching. MSE loss function can be expressed as follows:
  (4) $$\begin{array}{c} L_{\mathrm{MSE}}=\frac{1}{W\cdot H}{\left\|F\left(x_{\text{detail}}\right)-\left(x-y\right)\right\|}^{2}, \end{array}$$
where *x* is the noise image, *y* is the real CT image, and *W* and *H* are the width and height of input image to {*x*, *y*}, respectively.
(2) Perceptual loss function. The traditional MSE loss pixel-by-pixel comparison method often causes the loss of high-frequency information. A perceptual loss function is introduced to improve the denoising effect of the existing blur, realize edge enhancement, and enhance its texture details. By comparing the differences between image features, the perceptual loss can reconstruct more details and obtain better denoising effects. Experiments prove that the neural network used for image classification and segmentation can learn well the semantic features such as texture edges of images. The pretrained convolutional networks, therefore, can be connected in series to extract the required feature maps.

SegNet model comprising a set of convolutional coding layers and mirrored deconvolutional decoding layers can achieve better effect in semantic segmentation and thus is selected for the loss network. The encoding part uses the visual geometry group (VGG) model with strong generalization ability, and the decoding part uses a symmetrical structure to recover the information lost in pooling. Besides, the pretrained Caffe model is used to ensure the ability of the loss network to extract features.

After determining the loss network, perceptual loss needs to be defined at the semantic feature level. The specific steps are as follows: input the fuzzy denoising result *x* − *F*(*x*_detail_) and real image *y* initially generated by the front-end network into SegNet. The feature maps of these two are extracted from the fixed convolutional layer, and then the Euclidean distance represented by these two features is calculated, as shown in the following equation:

(5) $$\begin{array}{c} L_{\mathrm{Per}}=\frac{1}{W_{i}H_{i}}{\left\|\varphi_{i}\left(x-F\left(x_{\text{detail}}\right)\right)-\varphi_{i}\left(y\right)\right\|}^{2}, \end{array}$$

where *W*_*i*_ and *H*_*i*_ represent the width and height of the selected feature map, respectively, and *φ*_*i*_ is the feature map extractor.

The joint perceptual loss consists of two parts, namely MSE and perceptual loss. The structural model is shown in Figure 3. The method is implemented as follows: first, noisy CT image and real CT image *y* are input into the denoising network. The difference between these two is compared and learned pixel by pixel through the MSE loss function, and the initial denoising result *x* − *F*(*x*_detail_) that matches pixel *y* is obtained. At this time, the CT image after initial denoising is blurry. On this basis, *y* and *x* − *F*(*x*_detail_) are input into the loss network SegNet, respectively. Then the two feature maps *φ*(*x* − *F*(*x*_detail_)) and *φ*(*y*) are extracted from one of the convolutional layers to define the perceptual loss function. The network continues to train by minimizing perceptual loss to learn the difference in semantic features of these two images, reconstruct the edge and detail information, and make the two images more similar in feature perception. Finally, a clearer CT image denoising result is generated.

### 3.4. Optimization Process

The signal-to-noise ratio of CT images after training on the RED-CNN is significantly improved. To further eliminate the residual artifact noise of CT images, improve its detailed texture, and achieve a better correction effect, CT noise images generated by the RED network are processed by tissue processing technology based on clustering segmentation.

The residual artifact noise is weak. In the process of neural network training, this part of artifact noise is not obvious enough, so it is difficult for the network to accurately identify and remove it. To clear all the residual noise in CT images, there is a need to process the water equivalent tissue. Given that water equivalent tissues are similar in X-ray attenuation and dominate images, a uniform value must be assigned to these pixels so as to clear the residual metal artifacts in flat areas.

Firstly, the k-means clustering segmentation principle is followed, and CT images are automatically segmented into three parts: bone, water (including water equivalent tissue), and air based on two thresholds. To avoid clustering errors, the bone-water threshold is set to be no less than 320 HU. On this basis, the image after cluster segmentation is transformed into a binary image. Among them, the water pixel is 1, and the remaining pixels are 0. However, when the water pixel area is a constant value, a false boundary or structure will appear as a result of discontinuity in boundary data. Therefore, based on the calculation of the distance between two pixels, a transition area of *L* *=* *5* pixels is set in the water pixel area. If the distance between the pixel and its nearest 0 pixel is greater than *L*, the pixel value is set to *L*; otherwise, it is set to distance *D* between the two. The weighted average of water pixels for optimized images of the image trained by the neural network is shown in the following equation:

(6) $$\begin{array}{c} {\overset{-}{y}}^{\text{Net},w}=\frac{\sum_{i}D_{i}y_{i}^{\text{Net}}}{\sum_{i}D_{i}}. \end{array}$$

Furthermore, the prior image is obtained as shown in the following equation:

(7) $$\begin{array}{c} y_{i}{}^{\text{prior}}=\frac{D_{i}}{L}{\overset{-}{y}}^{\text{Net},w}+\left(1-\frac{D_{i}}{L}\right)y_{i}^{\text{Net}}. \end{array}$$

In the algorithm, RED-CNN training and optimization are two mutually beneficial steps. CT images trained by the RED-CNN can eliminate most artifact noise. On this basis, the residual fine artifact noise is further eliminated, and misclassification is avoided combined with optimized processing technology. In this paper, the transition area of water equivalent organization is added to the optimization processing link to eliminate the data discontinuity caused by the same threshold allocation. When a clear and accurate edge structure is restored, the residual artifact noise in the area is cleared, and the generated images attain a higher signal-to-noise ratio.

## 4. Experiment and Analysis

The hardware environment of the experimental platform is as follows: the operating system is Windows 10, central processing unit (CPU) is Intel Core i7-1065G7, and the graphics card model is Radeon Graphics 8 core. TensorFlow deep learning framework is used to perform denoising tests on CT images from the TCGA-COAD clinical data set. The experiment selects 200 different CT images with a size of 512 × 512 pixels as training data. LDCT images in the experiment can be simulated by adding noise to the NDCT image projection domain.

### 4.1. Experimental Parameters and Evaluation Indicators

The experimental parameters of the CT image denoising algorithm based on the RED network are set as follows: the size of the image block is 48 ∗ 48, the learning rate *α* = 10^−5^, and the number of cycles *S* *=* *5*. The number of layers in the encoder-decoder network is 8; the number of convolution kernels in the last layer is 1; the number of other layers is 64; and the convolution kernels in all layers have a size of 3 ∗ 3. The step size of convolution and deconvolution is set to 1 without zero padding. The convolution and deconvolution kernels are initialized with a random Gaussian distribution with a mean value of 0 and a standard deviation of 0.01. The network saves parameter information every 1,000 training, and terminates training after 50,000 iterations.

In order to better evaluate the denoising effect of the algorithm on noisy CT images, quantitative evaluation indexes of peak signal-to-noise ratio (PSNR) and structural similarity (SSIM) are introduced [29, 30]. The two evaluation indicators are defined as follows:

(1) PSNR:
  (8) $$\begin{array}{c} \text{PSNR}=20\;\log_{10}\frac{255}{\sqrt{1/mn\sum_{i=0}^{m-1}\sum_{j=1}^{n-1}{\left[I\left(i,j\right)-K\left(i,j\right)\right]}^{2}}}, \end{array}$$
where *I* is the real CT image of *m* × *n* and *K* is the CT image after noise removal.
(2) SSIM:
  (9) $$\begin{array}{c} \text{SSIM}=\frac{\left(2\mu_{x}\mu_{x^{\prime }}+c_{1}\right)\left(2\sigma_{xx^{\prime }}+c_{2}\right)}{\left(\mu_{x}^{2}+\mu_{x^{\prime }}^{2}+c_{1}\right)\left(\sigma_{x}^{2}+\sigma_{x^{\prime }}^{2}+c_{2}\right)}, \end{array}$$
where *μ*_*x*_ and *μ*_*x*′_ are the mean values of images *x* and *x′*, respectively, and *σ*_*x*_ and *σ*_*x*′_ are the standard deviations of images *x* and *x′*, respectively. *σ*_*xx*′_ is the covariance of *x* and *x′*, and *c*_1_ and *c*_2_ are constants.

### 4.2. Convergence Analysis

As the network rises in depth, the model's accuracy will reach saturation and then degenerate rapidly, which makes convergence unattainable and cause the training accuracy of the network to decline. The residual network, however, can speed up the convergence of network loss function and solve the problem of gradient disappearance and degradation caused by the increase in the number of network layers.  Figure 4 shows the convergence speed of loss function for residual network and nonresidual network with the number of iterations. It can be seen from Figure 4 that compared to the nonresidual network, the residual network converges faster, and the loss value after convergence is smaller. This demonstrates that the residual learning has outstripped direct mapping in the learning effect, which can minimize the difference between input images and target images. The mapping after the introduction of residual is more sensitive to the change of output, which improves the model accuracy while maintaining the depth of the network.

The performance of the training model is determined by the number of layers of neural network and residual units. In order to further determine the appropriate number of residual network layers and residual units, this paper has trained and tested the network with the number of layers at 4, 8, and 12 and the number of residual units at 2, 3, and 4, respectively.  Table 1 shows the average time required for different network models to iterate once under the same training set. As can be seen from Table 1, the 8-layer RED network iteration takes 247.349 s, which is shorter in time and faster in training speed.

This paper selects hip joint prosthesis as the test set to evaluate the image quality of the network after training with the number of layers at 4, 8, and 12, respectively.  Table 2 shows SSIM value, RMSE value, and PSNR value of images after three network training. As can be seen from Table 2, when the number of RED network layers is 8, the output image shows a better evaluation index: a larger SSIM value, a smaller RMSE value, and a larger PSNR value, which indicate that the network has a higher performance in image restoration. In summary, when the network model has 8 layers, it can achieve faster convergence speed, higher image quality after correction, and better performance of metal artifact correction.

### 4.3. Subjective Effects

Nine CT images were randomly selected from the TCGA-COAD clinical data set as test charts. It does not overlap with 200 images used for training, as shown in Figure 5. This paper selects the WGAN algorithm proposed in reference [23] and the basic RED-CNN algorithm proposed in reference [28] as the comparison method.  Figure 6 shows the denoising effect by taking the test chart (a) and test chart (c) of Figure 5 as examples.

WGAN and basic RED-CNN are very similar to the proposed improved RED-CNN in subjective visual effects after denoising. However, after careful observation of these pictures, it is found that our proposed network is slightly better than the two in terms of detail retention.

### 4.4. Objective Indicators

For quantitative analysis, PSNR and SSIM are used to evaluate the denoising effect of LDCT images. Detailed data of the test chart are shown in Table 3. As can be seen from Table 3, our proposed method outperforms WGAN and basic RED-CNN in eight test images in objective indicators. The averaged PSNR is 1.865 dB, higher than that of the WGAN method, and 1.174 dB, higher than that of the RED-CNN method. SSIM is slightly ahead of WGAN in terms of indicators.

### 4.5. Complexity Comparison

The network complexity *E* can be defined by the following equation:

(10) $$\begin{array}{c} E=O\left\{\underset{l}{\sum }n_{l-1}f_{l}^{2}n_{l}\right\}n_{l}, \end{array}$$

where *n*_*l*_ is the number of feature maps output by the *l* layer of the network and *f*_*l*_ is the size of the *l* layer convolution kernel.

By calculating the average time consumption of 30 forward propagation for each test chart, the average CPU time consumption data is obtained. By calling the Caffe interface in python, the average GPU time consumption is obtained, as shown in Table 4.

Table 4 demonstrates that RED-CNN can save 40% of the time compared to WGAN. At the same time, the proposed method reduces the complexity of the algorithm through the notion of recursion, speeds up the convergence speed compared with the original RED-CNN, and reduces the time consumption by 75% compared with WGAN. Furthermore, it has better performance on GPU.

## 5. Conclusion

Due to the difficulty of modeling statistical features in the image domain, the existing methods of directly processing reconstructed images cannot eliminate image noise while maintaining image structure details. Deep learning offers great potential for the research in noise artifact restoration of LDCT images. In an attempt to overcome the problems of poor denoising performance for traditional algorithms, complex network model, and difficulty in training, this paper proposes a CT image denoising method based on an improved RED network. It is mainly divided into three parts: (1) the RED network is used to restore noisy CT images, and the notion of recursion is integrated into the RED network to reduce network complexity and boost operation efficiency; (2) with the advantages of MSE loss function and perceptual loss function combined, a joint loss function is proposed, and the edge and detail information are reconstructed through pixel-by-pixel comparison and minimizing the difference in image semantic features; and (3) the CT noise images generated by the RED network based on clustering segmentation technology are optimized to further suppress the artifacts and restore details. As shown in experimental simulation analysis of the TCGA-COAD clinical data set, the proposed method can generate higher PSNR and SSIM when compared with the WGAN method and original RED-CNN method. Furthermore, our method is low in algorithm complexity and can be well adapted to practical applications.

In the future, our proposed method is applicable to scenarios involving noise suppression, structure preservation, damage detection, and so on.

## Figures and Tables

**Figure 1:** Overall architecture of RED-Net with *S* stage recursion.

**Figure 2:** The architecture of shallow RED-Net.

**Figure 3:** Proposed joint loss of cascaded network.

**Figure 4:** Loss function of residual network and nonresidual network.

**Figure 5:** Experimental data.

**Figure 6:** Denoising results comparison images. (a) Original CT image. (b) Low-dose CT image. (c) WGAN. (d) RED-CNN. (e) Proposed algorithm.

**Table 1:** The average training time for 1 epoch of RED-CNN with the number of layers at 4, 8, and 12.

Network layers	Training time (s)
4	452.287
8	247.349
12	873.374

**Table 2:** SSIM, RMSE, and PSNR values under RED-CNN with the number of layers at 4, 8, and 12.

Network layers	SSIM	RMSE	PSNR
4	0.9584	0.0065	68.625
8	0.9592	0.0062	68.634
12	0.9576	0.0067	68.612

**Table 3:** PSNR and SSIM in experiments.

Number	Index	LDCT image	WGAN [23]	RED-CNN [28]	Proposed algorithm
*a*	PSNR/dB	25.375	28.346	28.783	30.245
	SSIM	0.768	0.912	0.921	0.942

*b*	PSNR/dB	24.653	26.398	29.012	29.374
	SSIM	0.731	0.892	0.901	0.911

*c*	PSNR/dB	24.987	29.321	30.876	31.238
	SSIM	0.763	0.924	0.932	0.953

*d*	PSNR/dB	23.826	27.873	28.987	30.872
	SSIM	0.711	0.865	0.912	0.934

*e*	PSNR/dB	30.145	32.146	31.273	31.698
	SSIM	0.863	0.962	0.920	0.925

*f*	PSNR/dB	27.836	30.124	30.023	30.836
	SSIM	0.792	0.845	0.823	0.912

*g*	PSNR/dB	26.834	29.834	29.867	31.345
	SSIM	0.723	0.835	0.844	0.902

*h*	PSNR/dB	26.214	30.013	29.839	31.314
	SSIM	0.719	0.862	0.843	0.909

*i*	PSNR/dB	22.245	26.215	27.831	30.134
	SSIM	0.712	0.821	0.873	0.901

Average	PSNR/dB	25.791	28.919	29.610	30.784
	SSIM	0.75	0.876	0.885	0.916

**Table 4:** Computational complexity comparison.

Parameter	WGAN	RED-CNN	Proposed algorithm
Complexity	3,713,000	2,703,000	2,383,000
Time/s(CPU)	15.923	8.344	3.921
Time/s(GPU)	6.213	2.981	0.352

## Data Availability

The data included in this paper are available without any restriction.
